RETRACTED

# Expression of MiR-608 in Nonsmall Cell Lung Cancer and Molecular Mechanism of Apoptosis and Migration of A549 Cells

**DOI:** 10.1155/2020/8824519

**Published:** 2020-12-22

**Authors:** Chu Huang, Weiming Yue, Lin Li, Shuhai Li, Cun Gao, Libo Si, Lei Qi, Chuanle Cheng, Ming Lu, Hui Tian

**Affiliations:** Department of Thoracic Surgery, Laboratory of Basic Medical Sciences, Qilu Hospital, Cheeloo College of Medicine, Shandong University, Jinan 250012, China

## Abstract

**Objective:**

This Work is aimed at exploring the effect of microRNA (MiR)-608 on the function of nonsmall cell lung cancer (NSCLC) A549 cells and related mechanisms.

**Methods:**

Blood samples of 106 NSCLC patients (experimental group) as well as 124 normal people (control group) were selected for relevant investigation. Polymerase chain reaction (PCR) as well as DNA sequencing was used to determine the genotyping of the MiR-608 rs4919510 polymorphism. MiR-608 expression in cells was detected by real-time PCR technology. Western blotting was used to detect changes in protein levels. NSCLC tissues as well as adjacent tissues were explored in 33 patients undergoing surgery.

**Results:**

MiR-608 rs4919510 does not influence the incidence of NSCLC patients. In addition, MiR-608 expression was downregulated in the tumor tissue of NSCLC patients, while the transcription factor activating enhancer-binding protein 4 (TFAP4) expression was upregulated. MiR-608 promotes DOX- (Doxorubicin-) induced apoptosis by negatively regulating TFAP4 expression in NSCLC tissue. TFAP4 can significantly inhibit the migration of A549 cells.

**Conclusion:**

The findings in this investigation can contribute to the effective treatment of NSCLC patients. Also, the investigation can provide some theoretical support for the application of new targets for NSCLC treatment.

## 1. Introduction

Lung cancer is a kind of malignant tumor. It is very harmful to human health as well as life [1]. Its morbidity and mortality have the fastest growth. 50 years ago, in many countries, it was reported that the number of lung cancer patients increased rapidly. In addition, its mortality rate also continued to increase. Among male patients, it is in the first place in all malignant tumors. Female morbidity ranks second [2, 3]. Lung cancer includes small cell lung cancer as well as nonsmall cell lung cancer (NSCLC). 85% to 90% lung cancers are NSCLC, which become the most common cause of cancer death [4]. Also, lung adenocarcinoma takes the largest proportion of all NSCLC [5]. At present, there is no clear conclusion about the cause and mechanism of lung cancer. Therefore, in addition to environmental carcinogenic factors, there are other unknown reasons for the extremely high morbidity of lung cancer. But it is mainly related to air pollution, tobacco exposure, and the conditions of the biological natural environment. MicroRNA (miRNA) is a large kind of endogenous noncoding single-stranded small molecule RNAs discovered in recent years. Many investigations have proved that miRNA is inextricably linked to the occurrence of cancer. Hao et al. (2017) reviewed the role of ectopic miRNAs in gastric cancer growth, migration, invasion, and apoptosis.

RETRACTED

Also, in terms of gastric cancer diagnosis as well as treatment, they paid attention to the application of abnormally expressed miRNA, which was taken as a potential biomarker.

The role of miRNA in gastric cancer can give a new research direction to tumorigenesis and development, as well as may become a new anticancer target [6]. Kulkarni et al. (2019) introduced the current understanding of miRNA exosome transmission and crosstalk as well as its downstream results, which finally results in cancer progression as well as metastasis. They discussed how exosome miRNAs give new targets to the cancer's treatment as well as detection [7].

The relationship between miRNA and NSCLC has been well studied. Dong et al. (2019) evaluated the potential of RNA Kcnq1ot1 in the progression of NSCLC. It was proved that the Kcnq1ot1 level was upregulated in NSCLC tissues as well as cell lines. Also, the reason for the high-level Kcnq1ot1 was the low overall survival as well as progression-free survival in NSCLC patients. In addition, in the development of NSCLC, through the axis of miR-27b-3p/HSP90AA1, Kcnq1ot1 plays the role of oncogene [8]. Liu et al. (2018) found that miRNA-1253 was obviously downregulated in NSCLC tissues. What is more, there is a correlation between it and late clinical stage, lymph node metastasis, and poor survival. In mouse subcutaneous tumors and metastatic NSCLC models, miRNA-1253 had the effect of inhibiting NSCLC in vivo [9]. Yin et al. (2017) explored the miRNA-221 role as well as potential mechanism in NSCLC through functional gain as well as loss analysis. It was found that compared with normal tissues and cells, the miRNA-221 expression was significantly lower than that in NSCLC tissues as well as cells. It suggests that as for the NSCLC treatment, miRNA-221 inhibition may be a potential target [10].

Although the relationship between miRNA and NSCLC has been well studied, the relationship between MiR-608 and NSCLC remains unclear. There are few researches about the relationship between MiR-608 and NSCLC. Therefore, MiR-608 is explored. In addition, the molecular mechanism of apoptosis and migration of A549 cells was investigated to provide a new target for NSCLC treatment. The MiR-608 rs4919510 polymorphism site is currently one of the most important MiR-608 single nucleotide polymorphisms reported to date. Therefore, the correlation of MiR-608 rs4919510 polymorphism site with NSCLC is mainly explored.

RETRACTED

## 2. Method

### 2.1. Research Sample

The samples used were all from Qilu Hospital. Blood samples were obtained from 106 NSCLC patients (experimental group) as well as 124 normal people (control group). There were no significant differences in age, height, and weight in the two groups of people in physical examination of the same period. Also, the correlation of the genotyping of MiR-608 rs4919510 polymorphism with NSCLC of these blood samples was determined. 33 patients undergoing surgery were screened out, to obtain the patients' NSCLC tissues as well as adjacent tissues. All patients underwent surgery in the Qilu hospital and did not undergo radiotherapy or chemotherapy. Patients and their family members were aware of the research content and signed informed consent. In addition, the research was approved by the hospital ethics committee. To avoid the influence of regional factors, all patients were from the Shandong province and its surrounding regions. Also, the patients had no relative relationship with each other. The apoptosis of human lung adenocarcinoma A549 cells was analyzed as well as divided into the control group, blank control group, MiR-608-C group, and MiR-608-G group. In the control group, it was necessary to treat the cells with DOX (Doxorubicin), while in the blank control group, it was only necessary to stain the cells. In groups of MiR-608-C as well as MiR-608-G, the DOX treatment was carried out while synthesizing exogenous MiR-608 to enhance its expression. In the experiment that TFAP4 promoted DOX-induced apoptosis in A549 cells, there were three groups, which were the control group, blank control group, and TFAP4 group. In the control group, it was necessary to treat the cells with DOX, while in the blank control group, it was only necessary to stain the cells, and in the TFAP4 group, DOX treatment was carried out while knocking down TFAP4.

### 2.2. Cell Culture

Roswell Park Memorial Institute (RPMI) 1640 (Gibco) as well as Dulbecco's Modified Eagle Medium (DMEM) (Gibco) was applied to the cultivation of human lung adenocarcinoma A549 cells as well as HEK-293 cells, respectively. All medium needed to be added with 10% fetal bovine serum (Shanghai Huiying Biotechnology Co., Ltd.), 100 U/mL penicillin, and 100 mg/mL streptomycin (Gibco). Then, it was necessary to put them into an incubator. The environment of the incubator should be 37°C and 5% CO_2_. Then, in terms of the subsequent experiments, cells in the logarithmic growth phase should be taken.

RETRACTED

The cell culture steps are as follows:

1. Cells frozen in liquid nitrogen at -196°C must be quickly thawed to 37°C to rapidly melt ice crystals frozen outside the cell to avoid the ice crystals slowly entering the cell to form recrystallization and causing damage to the cells
2. The old culture medium was carefully aspirated and washed (rinsed) with PBS (phosphate buffer saline). An appropriate amount of digestive juice (trypsin solution) was added. The amount of digestive juice was best to cover the cells. The optimal digestion temperature was 37°C
3. An inverted microscope should be applied to the observation of the digested cells. The contraction of cytoplasm as well as the disconnection of cells to pieces proves that the cells are digested properly at this time. The trypsin solution was discarded. It was noted to replace the pipette and add a fresh culture medium
4. The digested cells were pipetted into a cell suspension with a dropper. The cell suspension was aspirated into a 10 mL centrifuge tube. After equilibration, the centrifuge tube was placed in a tabletop centrifuge at 1000 rpm for 6-8 min. The supernatant was discarded. Then, it was necessary to add 2 mL culture solution, and the cells were gently pipetted with a dropper to make a cell suspension. According to the experimental requirements, cells were passaged or frozen

### 2.3. Genotyping

Polymerase chain reaction (PCR) as well as DNA sequencing was applied when genotyping was carried out. The blood samples of the people involved in the experiment were subjected to the extraction of blood genomic DNA, which was used in the detection of the MiR-608 rs4919510 polymorphism genotyping. Blood Mini Kit (Qiagen, Valencia, A) was applied to the blood genomic DNA extraction. Genomic DNA was a template. In addition, PCR was applied to the amplification of the target band. Finally, the genotyping was determined by DNA sequencing.

### 2.4. PCR Sequencing

The sample RNA extraction steps are as follows:

1. It was necessary to take and put the cryopreserved lysed cells at room temperature for 5 min. In this way, they could be completely dissolved
2. Two-Phase Separation: 0.2 mL of chloroform was added to the lysed sample by each 1 mL of Trizol reagent (Tiangen Biotech (Beijing) Co., Ltd.), and the tube cap was closed tightly. After vigorously shaking the tube manually for 15 s, it was incubated at 15 to 30°C for 2 to 3 min. It was centrifuged at 12000 rpm for 15 min at 4°C. After centrifugation, the mixed liquid would show the lower red phenol-chloroform phase, the middle layer, and the upper layer of the colorless aqueous phase where RNA was totally allocated. In terms of the aqueous phase volume, it was about 60% of the Trizol reagent added during homogenization
3. RNA Precipitation: The upper layer of the aqueous phase was put in a clean RNase-free centrifuge tube. It was necessary to add the isopropanol with equal volume and mix. In this way, the RNA can be precipitated. After incubation for 10 min at 15 to 30°C, it was centrifuged at 12000 rpm for 10 min at 4°C. At this time, RNA precipitation that was not visible before centrifugation formed a gel-like precipitation block on the bottom and side walls of the tube
4. RNA Cleaning: The supernatant was removed. At least 1 mL of 75% ethanol (75% ethanol prepared with DEPC (diethyl pyrocarbonate) (Takara Co., Japan) water) was added to each sample lysed by the 1 mL Trizol reagent to wash the RNA precipitation. After mixing, it was centrifuged at 7000 rpm for 5 min at 4°C
5. RNA Drying: Most of the ethanol solution was carefully aspirated to dry the RNA precipitation in room temperature air for 5-10 min
6. Dissolving RNA Precipitation: When dissolving RNA, 40 *μ*L of RNase-free water was first added and blown repeatedly with a gun several times to completely dissolve it. The obtained RNA solution was stored at -80°C until use

cDNA synthesis:

1. In terms of all cDNA samples, it was necessary to configure the real-time PCR reaction system separately. The solution was mixed by flicking the bottom of the tube and centrifuged briefly at 6000 rpm
2. The mixed solution was dried in a bath at 70°C for 3 min before adding reverse transcriptase. Immediately after taking out, the ice-water bath was performed until the temperature inside and outside the tube was consistent. Then, 0.5 *μ*L of reverse transcriptase was added and it was placed in a 37°C water bath for 60 min
3. Immediately after taking out, it was dried in a bath at 95°C for 3 min. The final reverse transcription solution was the cDNA solution. It was necessary to put it at -80°C to standby

RETRACTED

### 2.5. Real-Time PCR

As far as real-time PCR technology is concerned, in the PCR reaction system, fluorescent groups were added. In addition, the entire PCR process was monitored by fluorescence signal accumulation in real-time, and then quantitative analysis was carried out on the unknown template by using a standard curve [11].

q-RT PCR sample detection:

1. In terms of all cDNA samples, it was necessary to configure the real-time PCR reaction system separately
2. The obtained real-time PCR reaction system was centrifuged at 6000 rpm briefly
3. The prepared PCR reaction solution was placed on a real-time PCR instrument (Bio-Rad Company, USA) to perform a PCR amplification reaction. The reaction should be carried out under the following environment. It was necessary to carry out the predenaturation at 93°C for 2 min; then, according to 93°C for 1 min, 55°C for 1 min, and 72°C for 1 min, 40 cycles in total were performed; finally, the extension was performed at 72°C for 7 min

### 2.6. Cell Transfection

The steps of cell transfection are as follows:

1. Preparation of Transfection Reagent: 400 *μ*L of nuclease-free water was added to the tube and shaken for 10 s to dissolve the fat. After shaking, the reagent was stored at -20°C, and it needed to be shaken before use
2. The appropriate mixing ratio (1 : 1-1 : 2/liposome volume: DNA quality) was selected to transfect the cells. An appropriate volume of serum-free medium was added to a transfection tube. DNA of MyoD (Myogenic Differentiation Antigen) (Wuhan Chundu Biotechnology Co., Ltd.) or EGFP (Enhanced Green Fluorescent Protein) (Beijing Biocytogen Co., Ltd) of appropriate quality was added. After shaking, the appropriate volume of transfection reagent was added and it was shaken again
3. The mixed solution was placed at room temperature for 10-15 min
4. The medium from the culture plate was aspirated and washed once with PBS or serum-free medium
5. After the mixed solution was added, the cells were put back into the incubator for 1 h
6. Whether to remove the mixed solution was decided according to the type of cells. Then, a complete medium was added to continue culturing for 24-48 h

### 2.7. Apoptosis Experiment

Doxorubicin (DOX) (Sigma Inc., USA) is a first-line clinical cancer treatment drug widely used to treat a variety of malignant tumors. In terms of the transcription factor activating enhancer-binding protein 4 (TFAP4), it is a significant regulator, which plays an essential part in cancer occurrence as well as development [12, 13].

It was necessary to wash the normally cultured as well as induced suspension cells (0.5 ~ 1 × 106) by PBS. 100 *μ*L Binding Buffer as well as 10 *μ*L Annexin-V (Shanghai Yeasen Biotech Co., Ltd.) (20 *μ*g/mL) labeled by FITC (fluorescein isothiocyanate) was added at room temperature in the dark for 30 min. Then, 5 *μ*L PI (propidium iodide) (Shanghai Haoran Biological Company) (50 *μ*g/mL) was added. After reacting in the dark for 5 min, 400 *μ*L Binding Buffer was added. Immediately, FACScan (Fluorescence Activating Cell Sorter) was used for quantitative detection by flow cytometry.

24 h after transfection, it was necessary to treat the cells by applying DOX with different concentrations for 24 h according to different groups, followed by trypan blue staining.

4% trypan blue mother liquor (Shanghai Hengyuan Biological Technology Co., Ltd.) was diluted to 0.4% with PBS solution and put in a 37°C water bath to preheat. Trypsin digested adherent cells to prepare a single-cell suspension, and it was diluted appropriately. The cell suspension and trypan blue staining solution were mixed in a ratio of 9 : 1, and the final solution concentration was 0.04%. The cells were counted under the microscope. The cell viability was counted, as shown in the following equation.

(1) $$\begin{array}{c} \text{Cell mortality rate }\left(\%\right)=\text{Number of dead cells}/\text{Total number of cells}\times 100\%. \end{array}$$

RETRACTED

### 2.8. Western Blotting

Western blotting is to transfer proteins to the membrane as well as apply antibodies to detection [14]. As far as the known expressed protein is concerned, it was necessary to apply the primary antibody to the detection of the corresponding antibody. Moreover, it was necessary to apply the antibody of the fusion part in the detection of the expression product of the new gene [15]. Cells in each group were lysed by RIPA lysate (1 mL RIPA (Radio Immunoprecipitation Assay) +10 *μ*L PMSF (phenylmethanesulfonyl fluoride) +10 *μ*L aprotinin) for 30 min and operated on ice. It was collected in an Eppendorf tube.

As for the determination of protein concentration, it was necessary to apply BCA (bicinchoninic acid) protein quantitative method. The protein sample per lane was 10 *μ*g. After the separation of 10% SDS-PAGE (Sodium dodecyl sulphate polyacrylamide gel electrophoresis), it was necessary to put the protein into PVDF (polyvinylidene fluoride) (Millipore, USA) membrane by the wet method. Also, it was blocked with PBST (phosphate-buffered solution) containing 5% bovine serum protein (Gibco, USA) for 1 h. Then, it was necessary to add the corresponding I antibody as well as incubate it overnight at 4°C. After washing the membrane 3 times with TBST (Tris-HCl buffered saline solution+Tween) (Beijing Solarbio Science & Technology Co., Ltd.), it was necessary to add the corresponding II antibody as well as incubate it at room temperature for 2 h. After that, it was necessary to wash the membrane 3 times by applying TBST as well as ECL (electrochemiluminescence) luminescence kit (Beijing Ruier Xinde Technology Co., Ltd.) was used for luminescence development. An analysis was conducted after fixing.

### 2.9. Statistical Method

SPSS 26.0 software was applied to the data processing. Mean ± standard deviation was applied to the expression of continuous variables. One-way analysis of variance was applied to the comparison between groups. When the variances are equal, the *t* test is used. When the variances are unequal, the *t* test is used. *P* < 0.05 indicates that the difference is statistically significant, while *P* < 0.01 indicates that the difference is significantly statistically significant.

RETRACTED

## 3. Results and Discussion

### 3.1. MiR-608 rs4919510 Polymorphic Site and NSCLC

Determining the correlation between the MiR-608 rs4919510 polymorphism site and NSCLC is the first step in this investigation.  Figure 1 shows the results obtained.

As can be seen from Figure 1(a), in the normal population, 24.3% of people belonged to the CC genotype, 41.9% of people belonged to the CG genotype, and 33.8% of people belonged to the GG genotype. In patients with NSCLC, the CC genotype accounted for 19.7%, the CG genotype accounted for 47%, and the GG genotype accounted for 33.3%. No significant difference can be seen between the two groups (*P* > 0.05). As can be seen from Figure 1(b), in all normal populations, the C allelic gene accounted for 45.2%, and the G allelic gene accounted for 54.8%. In all patients with NSCLC, the C allelic gene accounted for 43.2%, and the G allelic gene accounted for 56.8%. No significant difference can be seen between the two groups (*P* = 0.608 > 0.05).

### 3.2. Expression of MiR-608 in NSCLC Tissue

MiR-608 expression levels in lung cancer tissues as well as adjacent tissues of 33 patients with NSCLC were detected.  Figure 2 shows the results.

Figure 2 reveals that the MiR-608 expression level in the cancer tissues of 27 NSCLC patients had a downward trend. Moreover, in terms of the average difference between cancer tissues and adjacent tissues, it was 2.6 times. The difference between the two was statistically significant (*P* < 0.05). Based on the above description and results, it can be reasonably speculated that MiR-608 is a tumor suppressor gene, which is of great significance in the occurrence as well as the development of NSCLC.

### 3.3. MiR-608 and A549 Cells

Whether the function of MiR-608 in A549 cells is changed by the polymorphism should be determined. Therefore, it was necessary to synthesize exogenous MiR-608-C as well as MiR-608-G. In this way, the MiR-608 expression in A549 cells could be enhanced. The results are shown in Figure 3. NC is the blank control group.

It can be seen from Figure 3 that the MiR-608 level of the MiR-608-C group and MiR-608-G group was significantly higher than that of the control group and blank control group. Although the MiR-608 level of the MiR-608-G group was higher than that of the MiR-608-C group, the difference was not obvious. The MiR-608 level between the control group and the blank control group was not obviously different. The MiR-608 expression level after the MiR-608 overexpression in A549 cells indicates that MiR-608-C as well as MiR-608-G will seriously affect the MiR-608 expression in A549 cells.

RETRACTED

The results of the influence of the MiR-608 overexpression alone on the apoptosis of A549 cells are shown in Figure 4.

As can be seen from Figure 4, although the ratio of death cell to apoptotic cell in MiR-608-C group, MiR-608-G group, control group, and blank control group was different, there was no obvious difference. Trypan blue staining and cell assay found no change in the level of cell death after the overexpression of MiR-608 in A549 cells. Therefore, MiR-608 overexpression alone has no obvious influence on A549 cell apoptosis.

The effect of MiR-608 on the cell apoptosis after DOX treatment of A549 cells was detected. The results are shown in Figure 5.

It can be seen from Figure 5 that the cleaved-caspase-3 level of MiR-608-C and MiR-608-G groups was significantly higher than that of the control and blank control groups; the cleaved-caspase-3 level of the MiR-608-G group was higher than that of the MiR-608-C group, but the difference was not obvious; the cleaved-caspase-3 level of the control group and the blank control group was not obviously different. After low-dose (0.2 *μ*M) DOX treatment of A549 cells, the overexpression of MiR-608 will result in an obvious increase in the cleaved-caspase-3 protein expression level. It indicates that the level of apoptosis of A549 cells has increased.

Also, Figure 6 depicts the apoptosis and cell death after low-dose (0.2 *μ*M) DOX treatment of A549 cells.

It can be seen from Figure 6 that the ratio of apoptotic cells induced by simple low-dose DOX was less than 10%. However, when MiR-608 was overexpressed in Dox-treated cells, the apoptosis rate of the MiR-608 overexpression group increased significantly. It indicates that MiR-608 overexpression increases the sensitivity of A549 cells to DOX drugs, which also indicates that MiR-608 has a function of proapoptotic in the NSCLC development.

### 3.4. MiR-608 Promoting DOX-Induced Apoptosis of A549 Cells by Regulating TFAP4

The results of TFAP4 promoting DOX-induced apoptosis of A549 cells are shown in Figure 7.

It can be seen from Figure 7(a) that with the passage of time, the TFAP4 mRNA level of A549 cells decreased significantly after 3 hours until it showed a steady state. After high-dose (0.2 *μ*M) DOX treatment of A549 cells, there was an obviously downward trend in TFAP4 mRNA expression level. As can be seen from Figure 7(b), the apoptosis rate of the TFAP4 group was significantly higher than that of the control group and the blank control group, and there was no significant difference between the two groups. After endogenous TFAP4 knockdown, A549 cells were treated with low-dose DOX, and the cell death increased significantly. It shows that TFAP4 will affect the sensitivity of A549 cells to DOX.

RETRACTED

As shown in Figure 8, it was further found that in the absence of DOX treatment, the overexpression of MiR-608 led to the decrease in TFAP4 protein expression. When cells were treated with high-dose DOX, TFAP4 levels decreased overall. The DOX and MiR-608 overexpression cotreatment group showed the most significant decrease in TFAP4.

### 3.5. TFAP4 Promoting Migration of A549 Cells

As can be seen from Figure 9, the cell migration rate of the TFAP4 group at 24 h was not significantly different from that of the control group and the blank control group; that of the TFAP4 group was significantly lower than the control group and the blank control group at 48 h. After knocking down TFAP4, the migration of A549 cells was inhibited. It shows that TFAP4 will have a certain effect on cell migration and can significantly inhibit A549 cell migration.

## 4. Discussion

Many investigations have proved that miRNA plays an important role in many diseases. In addition to oncogenes, miRNA is also a tumor suppressor gene. miRNA has a quite close relationship with the occurrence of cancer [16, 17]. Thus, miRNA and NSCLC are connected to study the correlation of miRNA-608, NSCLC, and with A549 cells.

After this investigation, there was no correlation of the rs4919510 polymorphism at the 4th position of MiR-608-3p and NSCLC. No significant difference could be seen in the rs4919510 genotype between the normal population and NSCLC patients. Thus, the MiR-608 expression in lung cancer tissues was explored. It was found that the MiR-608 expression in cancer tissues was obviously reduced compared to the adjacent tissues. The difference between the two was as much as 2.6 times, which shows that there is a certain relationship between MiR-608 and NSCLC. Wang et al. (2019) explored the effect of MiR-608 rs4919510 on the incidence of lung cancer patients. The results showed that the MiR-608 rs4919510 presence had no influence on the susceptibility of patients to NSCLC or the maturity of MiR-608, but the MiR-608 expression level in NSCLC tissues was downregulated. In addition, the overexpression of MiR-608 promoted apoptosis induced by NSCLC cell lines A549 as well as HCC4006 by inhibiting the expression of TFAP4 [18]. It is almost consistent with the results of the investigation. However, in this investigation, it was found that MiR-608 promotes DOX-induced apoptosis of A549 cells by regulating TFAP4. After high-dose DOX (2 *μ*M) treatment of A549 cells, TFAP4 expression level in mRNA decreased significantly [19, 20]. Also, TFAP4 can significantly inhibit the A549 cells' migration. Therefore, the results of this investigation may provide valuable insights for the chemotherapy of NSCLC.

RETRACTED

## 5. Conclusion

Due to the current uncertainty about the pathogenesis and cause of NSCLC as well as the high morbidity and mortality of NSCLC, MiR-608, which may be related to NSCLC, was explored. It was found that there was an inevitable link between MiR-608 and NSCLC. MiR-608 can promote DOX-induced apoptosis of A549 cells by regulating TFAP4. Although some results have been achieved, there are still some shortcomings. During the investigation, no joint research was conducted on the daily lives of the participants. At present, it is believed that lung cancer infection may be affected by age, gender, region, and smoking status. The above factors are not considered in the investigation. Therefore, in the next step, a more comprehensive investigation will be conducted to determine the specific correlation. Also, the clinical significance as well as the specific mechanism of TFAP4 and miR-608 in the progress of lung cancer needs further investigation.

## Figures and Tables

**Figure 1:** Correlation between MiR-608 rs4919510 polymorphism site and NSCLC ((a) proportion of genotypes in two groups; (b) proportion of allelic genes in two groups).

**Figure 2:** Results of detection of MiR-608 expression level ((a) MiR-608 expression level in all patients; (b) comparison of MiR-608 expression level in adjacent tissues as well as cancer tissues of patients).

**Figure 3:** MiR-608 overexpression level.

**Figure 4:** The results of the effect of the overexpression of MiR-608 alone on the A549 cell apoptosis.

**Figure 5:** The effect of MiR-608 on cell apoptosis after DOX treatment of A549 cells.

**Figure 6:** The apoptosis and cell death after low-dose (0.2 *μ*M) DOX treatment of A549 cells.

**Figure 7:** The results of TFAP4 promoting DOX-induced apoptosis of A549 cells ((a) TFAP4 mRNA expression level after high-dose DOX treatment of A549 cells; (b) A549 cell death after low-dose DOX treatment and TFAP4 knockdown).

**Figure 8:** TFAP4 protein expression.

**Figure 9:** The results of the effect of TFAP4 on the A549 cells' migration.

## Data Availability

All data, models, and code generated or used during the study appear in the submitted article.

## References

[1] Prat A., Navarro A., Paré L. (2017). Immune-related gene expression profiling after PD-1 blockade in non–small cell lung carcinoma, head and neck squamous cell carcinoma, and melanoma. *Cancer Research*.

[2] Lee C. K., Man J., Lord S. (2018). Clinical and molecular characteristics associated with survival among patients treated with checkpoint inhibitors for advanced non–small cell lung carcinoma: a systematic review and meta-analysis. *JAMA Oncology*.

RETRACTED

[3] Zappa C., Mousa S. A. (2016). Non-small cell lung cancer: current treatment and future advances. *Translational Lung Cancer Research*.

[4] Parra E. R., Villalobos P., Mino B., Rodriguez-Canales J. (2018). Comparison of different antibody clones for immunohistochemistry detection of programmed cell death ligand 1 (PD-L1) on non–small cell lung carcinoma. *Applied Immunohistochemistry & Molecular Morphology*.

[5] Sun Z., Shi K., Yang S. (2018). Effect of exosomal miRNA on cancer biology and clinical applications. *Molecular Cancer*.

[6] Hao N. B., He Y. F., Li X. Q., Wang K., Wang R. L. (2017). The role of miRNA and lncRNA in gastric cancer. *Oncotarget*.

[7] Kulkarni B., Kirave P., Gondaliya P. (2019). Exosomal miRNA in chemoresistance, immune evasion, metastasis and progression of cancer. *Drug Discovery Today*.

[8] Dong Z., Yang P., Qiu X. (2018). KCNQ1OT1 facilitates progression of non-small-cell lung carcinoma via modulating miRNA-27b-3p/HSP90AA1 axis. *Journal of Cellular Physiology*.

[9] Liu M., Zhang Y., Zhang J. (2018). MicroRNA-1253 suppresses cell proliferation and invasion of non-small-cell lung carcinoma by targeting WNT5A. *Cell Death & Disease*.

[10] Yin Z., Xu M., Li P. (2017). miRNA-221 acts as an oncogenic role by directly targeting TIMP2 in non-small-cell lung carcinoma. *Gene*.

[11] Xia H., Jing H., Li Y., Lv X. (2018). Long noncoding RNA HOXD-AS1 promotes non-small cell lung cancer migration and invasion through regulating miR-133b/MMP9 axis. *Biomedicine & Pharmacotherapy*.

[12] Lingzi X., Zhihua Y., Xuelian L. (2016). Genetic variants in microRNAs predict non-small cell lung cancer prognosis in Chinese female population in a prospective cohort study. *Oncotarget*.

[13] Zhang N., Li Y., Zheng Y. (2019). miR-608 and miR-4513 significantly contribute to the prognosis of lung adenocarcinoma treated with EGFR-TKIs. *Laboratory Investigation*.

[14] Jin Z., Jin R. H., Ma C., Li H. S., Xu H. Y. (2017). Serum expression level of miR-504 can differentiate between glioblastoma multiforme and solitary brain metastasis of non-small cell lung carcinoma. *Journal of BUON*.

[15] Yu H. X., Wang X. M., Han X. D., Cao B. F. (2018). MiR-608 exerts tumor suppressive function in lung adenocarcinoma by directly targeting MIF. *European Review for Medical and Pharmacological Sciences*.

[16] Othman N., Nagoor N. H. (2017). miR-608 regulates apoptosis in human lung adenocarcinoma via regulation of AKT2. *International Journal of Oncology*.

[17] Wang Y., Li F., Ma D., Gao Y., Li R., Gao Y. (2019). MicroRNA-608 sensitizes non-small cell lung cancer cells to cisplatin by targeting TEAD2. *Molecular Medicine Reports*.

RETRACTED

[18] Wang Y.-F., Ao X., Liu Y. (2019). MicroRNA-608 Promotes apoptosis in non-small cell lung cancer cells treated with doxorubicin through the inhibition of TFAP4. *Frontiers in Genetics*.

[19] Hendry S., Salgado R., Gevaert T. (2017). Assessing Tumor-Infiltrating lymphocytes in solid tumors. *Advances in anatomic pathology*.

[20] Heymann J. J., Bulman W. A., Swinarski D. (2017). PD-L1 expression in non-small cell lung carcinoma: comparison among cytology, small biopsy, and surgical resection specimens. *Cancer Cytopathology*.

